The article "The Clinical Efficacy of Tirofiban Combined with Ticagrelor and Aspirin in Treating Acute Myocardial Infarction by Percutaneous Coronary Intervention and Its Effect on Patients' Cardiac Function" was published in 2022. Journal: J Healthc Eng.

# The Clinical Efficacy of Tirofiban Combined with Ticagrelor and Aspirin in Treating Acute Myocardial Infarction by Percutaneous Coronary Intervention and Its Effect on Patients' Cardiac Function

**DOI:** 10.1155/2022/4708572

**Published:** 2022-02-09

**Authors:** Rui Peng, Feng Li

**Affiliations:** ^1^Department of Heart Center, The First Hospital of LanZhou University, LanZhou 730000, Gansu, China; ^2^Department of Internal Medicine-Cardiovascular, Xiang'an Branch, The First Affiliated Hospital of Xiamen University, Xiamen 361101, Fujian, China

## Abstract

**Objective:**

To explore the clinical efficacy of tirofiban combined with ticagrelor and aspirin in acute myocardial infarction treatment by percutaneous coronary intervention and its effect on patients' cardiac function.

**Methods:**

We selected 102 patients with acute myocardial infarction who came to The First Hospital of LanZhou University for treatment from July 2018 to May 2021. On the basis of conventional treatment, patients were separated into a joint group (tirofiban combined with ticagrelor and aspirin) comprising 55 cases and a control group (conventional ticagrelor and aspirin dual treatment) involving 47 cases. Blood flow classification of the two groups of patients was immediately recorded and compared after the myocardial infarction thrombolysis test (TIMI). Left ventricular function-related indicators, platelet-related parameters, neutrophil/lymphocyte ratio (NLR), red blood cell distribution width (RDW), and platelet/lymphocyte ratio (PLR) before treatment and 7 days after PCI were evaluated and compared between the groups before treatment and 3 months after treatment. ELISA was utilized to detect the serum levels of inflammatory factors, tumor necrosis factor-*α* (TNF-*α*), interleukin-6 (IL-6), and hypersensitive C-reactive protein (hs-CRP) before and after treatment. Incidence of major adverse cardiovascular events (MACEs) and adverse reaction incidence was put into comparison between the two groups in the course of the 3-month follow-up period. Compared with the control group, the joint group accounted for more patients with TIMI blood flow classification level 3 (*P* < 0.05) and showed more drastic improvement on the left ventricular function, platelet-related parameters, and serum inflammatory factors (*P* < 0.05). Moreover, patients of the joint group suffered less fluctuation from RDW, NLR, and PLR (*P* < 0.05), and their incidence of MACE was drastically lower in contrast with the control group (*P* < 0.05). No notable changes were presented in terms of incidence of adverse reaction (*P* > 0.05). For patients who suffered from acute myocardial infarction and treated with percutaneous coronary intervention, the application of tirofiban combined with ticagrelor and aspirin could effectively reduce the incidence of no reflow or slow blood flow, improve myocardial perfusion function, and have marked curative effects. It is worthy of clinical promotion and application.

The article "The Clinical Efficacy of Tirofiban Combined with Ticagrelor and Aspirin in Treating Acute Myocardial Infarction by Percutaneous Coronary Intervention and Its Effect on Patients' Cardiac Function" was published in 2022. Journal: J Healthc Eng.

## 1. Introduction

Acute myocardial infarction (AMI) is a cardiovascular disease with a high fatality rate caused by persistent myocardial ischemia and hypoxia, which can cause myocardial tissue necrosis and myocardial inflammation [1, 2]. For patients with AMI, an early opening of the infarct-related blood vessel is essential to determining the prognosis [3]. Percutaneous coronary intervention (PCI), an important method for infarction-related vascular reperfusion in patients with AMI in recent years, is currently widely regarded as one of the most efficient methods for AMI treatment, which can effectively relieve the obstruction and restore myocardial perfusion, thereby reducing the area of myocardial tissue necrosis and significantly improving the prognosis of patients to reduce the fatality rate [4, 5]. However, no reflow, slow blood flow, reperfusion arrhythmia, and acute thrombosis in the stent during operation increase the risks of related operation and postoperative treatment, so active antiplatelet therapy is extremely important [6].

As the drug of choice for antiplatelet therapy after coronary intervention, aspirin has a clear antiplatelet effect and has become the most widely used first-line antiplatelet drug [7]. Ticagrelor is a new selective P2Y12 receptor antagonist, which has a noncompetitive antagonistic effect on platelet aggregation induced by adenosine diphosphate [8]. But in recent years, with further research, more scholars believe that preoperative loading-dose dual antiplatelet therapy, also known as aspirin combined with P2Y12 receptor antagonist (ticagrelor), can effectively inhibit platelet aggregation and adhesion before emergency PCI [9]. As one of the conventional platelet GPIIb/III, a receptor antagonist, tirofiban has been found in the past to show good clinical effects in patients diagnosed with ST-segment elevation myocardial infarction (STEMI) undergoing emergency PCI, which can improve coronary blood flow, increase myocardial reperfusion, and help improve the efficacy [10]. Left ventricular ejection fraction (LVEF), left ventricular end-diastolic diameter (LVEDD), and left ventricular end-systolic diameter (LVESD) are currently more commonly used indicators of heart function assessment. Past studies have shown that patients with heart failure would have significant LVEDD, LVESD increase, and LVEF decrease. Therefore, it is also used as an index to evaluate a patient's cardiac function in this study.

The article "The Clinical Efficacy of Tirofiban Combined with Ticagrelor and Aspirin in Treating Acute Myocardial Infarction by Percutaneous Coronary Intervention and Its Effect on Patients' Cardiac Function" was published in 2022. Journal: J Healthc Eng.

These medications have different mechanisms of action. Therefore, it is believed that the combination of drugs can further obtain higher benefits through complementary mechanisms. However, information has existed currently about the use of tirofiban combined with ticagrelor and aspirin in the treatment of acute myocardial infarction in PCI. However, relatively few studies focused on the clinical efficacy of the disease. On the basis of that, this study proposes the use of tirofiban combined with ticagrelor and aspirin in patients with acute myocardial infarction undergoing PCI treatment, thereby providing more reference treatment options for antiplatelet therapy in patients with acute myocardial infarction. The results of this study also showed that tirofiban combined with ticagrelor and aspirin could bring more benefits to patients with acute myocardial infarction undergoing PCI treatment.

## 2. Materials and Methods

### 2.1. Clinical Information

We selected 102 patients diagnosed with AMI who came to The First Hospital of LanZhou University for treatment from July 2018 to May 2021. Based on the different treatment plans, patients were divided into a joint group (tirofiban combined with ticagrelor and aspirin) with 55 cases and a control group (conventional ticagrelor and aspirin dual treatment) with 47 cases. Inclusion criteria were as follows: patients diagnosed with AMI and met the indications for PCI; patients aged between 40 and 65 years old; and patients who agree to participate in the study. Exclusion criteria were as follows: patients with PCI contraindications; patients with severe coagulation dysfunction; patients with gastrointestinal bleeding; patients with severe organ dysfunction; patients who have undergone thrombolysis or warfarin before the onset; and patients with infectious diseases. All patients consented to the present study with a written informed form signed in person. This experiment has also been approved by The First Hospital of LanZhou University Ethics Committee and complies with the Helsinki Declaration.

### 2.2. Therapeutic Plans

All patients were given loading aspirin (Beijing Bayer Healthcare Co., Ltd., National Medicine Standard J20171021, specification: 0.1g) 300 mg chewed and ticagrelor (AstraZeneca Pharmaceutical Co., Ltd., National Medicine Standard J20171077, specification: 90 mg) 180 mg chewed, and unfractionated heparin 100 U/kg intravenously. On the basis of that, patients in the joint group were additionally given tirofiban injection (Ship Pharmaceutical Group Enbipu Pharmaceutical Co., Ltd., National Medicine Standard H20183440, specification: 100 ml and 5 mg). Initially, intravenous pumping was performed at a rate of 0.4 U/(kg·min) for 30 minutes. PCI was then performed after thrombolysis, followed by a postoperative intravenous pumping continuing at a rate of 0.1 U/(kg·min) for 24 to 36 hours. After the operation, both groups of patients were routinely given ticagrelor 90 mg twice a day and aspirin 100 mg once a day until 12 months after the operation. All patients were routinely treated with angiotensin-converting enzyme inhibitors, statins, calcium channel blockers, nitrates, and other drugs. Patients with other underlying diseases were given corresponding symptomatic treatment.

The article "The Clinical Efficacy of Tirofiban Combined with Ticagrelor and Aspirin in Treating Acute Myocardial Infarction by Percutaneous Coronary Intervention and Its Effect on Patients' Cardiac Function" was published in 2022. Journal: J Healthc Eng.

### 2.3. Observation Index

Immediately, the postoperative myocardial infarction thrombolytic test (TIMI) on the blood flow classification of two groups was recorded [12]. TIMI level 0: no forward blood flow at the distal end of the vascular occlusion; TIMI level 1: contrast agent partially passed through the occlusion site without filling the distal blood vessel; TIMI level 2: the contrast agent was able to fill the distal coronary artery completely but with a slower speed and lower clearance than the normal one; TIMI grade 3: the contrast agent could completely and rapidly fill and clear the distal blood vessels quickly.
(2) We compared the left ventricular function-related indicators of the two groups before treatment and 3 months after treatment, including left ventricular ejection fraction (LVEF), which refers to the percentage of heart stroke output to ventricular end-diastolic volume with the normal range of 50%–70%, left ventricular ejection fraction (LVEF) with the normal range of ventricular end-diastolic diameter (LVEDD) at 35–50 mm, and the normal range of left ventricular end-systolic diameter (LVESD) is 23–40 mm.
(3) An automatic blood cell analyzer (Beckman Coulter Co., Ltd., USA) was applied to detect the platelet-related parameters of two groups of patients after 30 days of treatment, including platelet volume distribution width (PDW), average platelet volume (MPV), platelet count (PLT), and platelet packed volume (PCT).
(4) We detected the platelet/lymphocyte ratio (PLR), neutrophil/lymphocyte ratio (NLR), and red blood cell distribution width (RDW) of two groups of patients before treatment and 30 days after PCI.
(5) The ELISA method was utilized to detect the serum inflammatory factor, tumor necrosis factor-*α* (TNF-*α*), interleukin-6 (IL-6), and hypersensitive C-reactive protein (hs-CRP) before treatment and 30 days after treatment.
(6) Incidence of major adverse cardiovascular events (MACEs), with cardiac death, severe heart failure (NYHA grade 3 and above), recurring myocardial infarction, and stent thrombosis included, were compared between two groups during the 3-month follow-up period.
(7) We recorded the incidence of adverse reactions among patients within 3 months of treatment for comparison, including general bleeding, massive hemorrhage, noncardiogenic dyspnea, and gastrointestinal reactions.

The article "The Clinical Efficacy of Tirofiban Combined with Ticagrelor and Aspirin in Treating Acute Myocardial Infarction by Percutaneous Coronary Intervention and Its Effect on Patients' Cardiac Function" was published in 2022. Journal: J Healthc Eng.

### 2.4. Statistical Methods

The SPSS 19.0 statistical software (Beijing Wangshu Times Technology Co., Ltd.) was applied for statistical analysis of the data, Prism 8 for statistical pictures required, case number and percentage (%) for count data, *χ*2 test for analysis, mean ± standard deviation for data measurement, paired *t* test for comparison before and after treatment, independent *t* test for comparison between two groups. The chi-square test was utilized, as shown in Tables 1–4, and independent *t* test and paired *t* test were utilized, as shown in Figures 1 and 2 and Tables 5 and 6. *P* < 0.05 indicated that the difference was statistically significant.

## 3. Results

### 3.1. General Information Comparison

Two groups of patients were comparable because of no notable discrepancies in terms of gender, age, BMI, and underlying diseases (*P* > 0.05), see Table 1 for details.

### 3.2. Comparison of Blood Flow Grading of Immediate Myocardial Infarction Thrombolysis Test (TIMI)

After treatment, the number of patients with grades 0, 1, 2, and 3 in the joint group was 0, 3, 10, and 42, respectively. That of those in the control group was 7, 10, 10, and 20, respectively. The proportion of patients in the joint group with TIMI grade 3 is significantly higher (*P* < 0.05), see Table 2 for details.

### 3.3. Comparison of Left Ventricular Function of Two Groups before and after 3 Months of Treatment

Before treatment, no notable difference was presented in LVEF, LVEDD, and LVESD (*P* > 0.05), while after 3 months of treatment, the LVEF of both groups was drastically higher than that before treatment, and both LVEDD and LVESD were notably lower than those before treatment, yet improvement in the joint group was more obvious when compared with the other group (*P* < 0.05), as is shown in Figure 1.

### 3.4. Comparison of Platelet-Related Parameters between Two Groups of Patients

Postoperative platelet count (PLT) of the joint group was smaller when compared with the control group, and its comparable numbers of platelet packed volume (PCT), mean platelet volume (MPV), and platelet distribution width (PDW) were all higher (*P* < 0.05), see Table 5 for details.

### 3.5. Comparison of Blood Cell-Related Parameters

There was no notable difference in platelet/lymphocyte ratio (PLR), red blood cell distribution width (RDW), and neutrophil/lymphocyte ratio (NLR) between the two groups before PCI surgery (*P* > 0.05), yet after PCI, RDW, NLR, and PLR of the two groups of patients on the 30th day were drastically different from those before surgery (*P* < 0.05), see Table 6 for details.

The article "The Clinical Efficacy of Tirofiban Combined with Ticagrelor and Aspirin in Treating Acute Myocardial Infarction by Percutaneous Coronary Intervention and Its Effect on Patients' Cardiac Function" was published in 2022. Journal: J Healthc Eng.

### 3.6. Comparison of Serum Inflammatory Factors before and after Treatment between Two Groups

Before treatment, no notable difference was shown in terms of serum hs-CRP, TNF-*α*, and IL-6 levels (*P* > 0.05). However, hs-CRP, TNF-*α*, and IL-6 of both groups underwent drastic declines after treatment (*P* < 0.05). Among which, a more notable reduction of indexes mentioned above showed in the joint group in contrast with the other one (*P* < 0.05), as shown in Figure 2.

### 3.7. The Incidence of MACE in the Two Groups of Patients

The number of people came down with cardiac death, recurrent myocardial infarction, severe heart failure, and stent thrombosis of the joint group were 0, 1, 1, and 1, respectively, with an MACE incidence rate of 5.45%. Numbers of those in the control group were 2, 3, 2 and 3, respectively, with a much higher incidence at 25.53%, indicating that the joint group had an obviously lower rate of MACE incidence (*P* < 0.05) (see Table 3 for details).

### 3.8. Comparison of Incidence of Adverse Reactions

The number of patients in the joint group who had general bleeding, hemorrhage, noncardiac dyspnea, and gastrointestinal reactions was 3, 0, 2, and 1, respectively, with an adverse reaction rate of 10.91%. Data referred in the control group were 2, 0, 1, and 1, respectively. The incidence of adverse reactions was around 8.51%, showing no drastic difference in adverse reaction incidence of two groups (*P* > 0.05) (see Table 6 for details).

## 4. Discussion

AMI mostly occurs in middle-aged and elderly patients, which is mainly due to the decline of systemic function, decreased vascular elasticity, and increased vascular stiffness which leads to increased pulse pressure in elderly patients [13]. If patients were not treated in time, it is likely to cause serious consequences because the opening of the infarct-related coronary artery and antiplatelet aggregation within the time window is the key to improving the prognosis of patients [14]. At present, the core treatment methods for AMI are reperfusion therapy and antithrombotic therapy [15]. Compared with drug therapy such as thrombolysis and anticoagulation, interventional therapy can significantly reduce the mortality of patients with AMI, and the choice of appropriate antiplatelet therapy is the cornerstone of interventional therapy. It is of great significance for opening blood vessels related to infarction, improving TIMI blood flow, reducing the incidence of no reflow or slow blood flow, reducing acute thrombosis in the stent, and reducing the incidence of severe heart failure and malignant arrhythmia attacks, and other MACE events [16, 17].

The article "The Clinical Efficacy of Tirofiban Combined with Ticagrelor and Aspirin in Treating Acute Myocardial Infarction by Percutaneous Coronary Intervention and Its Effect on Patients' Cardiac Function" was published in 2022. Journal: J Healthc Eng.

Ticagrelor is a fast-acting and reversible P2Y12 receptor antagonist. As a new type of adenosine diphosphate (ADP) receptor inhibitor, it enters the body with active ingredients and directly and reversibly binds to the P2Y12 receptor. The rapid inhibition of platelet aggregation has achieved good results in the interventional treatment of myocardial infarction [18]. Tirofiban is a new type of platelet GPIIb/III, a receptor antagonist that blocks the final pathway of platelet aggregation and inhibits thrombosis, which has a fast onset and a short half-life. Its effect would disappear within 3 to 5 hours after drug withdrawal, which can dissociate the aggregated platelets and recover the platelet function quickly. Once a bleeding event occurs, it is very helpful for drug adjustment and prevents the bleeding event from getting worse. Meanwhile, it can elevate the endothelial function of the body and facilitate myocardial perfusion. Tirofiban can also inhibit vasoconstriction to relax blood vessels, inhibit the release of inflammatory factors, and inhibit the release of oxygen free radicals from platelets [19, 20]. Aspirin, a nonsteroidal anti-inflammatory drug with good anti-inflammatory and antithrombotic effects, is mainly used clinically for primary and secondary prevention of arterial thrombosis [21]. However, there are relatively few clinical studies focused on the combined treatment of three medications mentioned at present. This is the first comprehensive analysis of the efficacy and safety of the combination of the three medications in patients with acute myocardial infarction treated by PCI. From the results of this study, the proportion of patients with the TIMI level III in the joint group was notably higher, indicating that the application of tirofiban combined with ticagrelor and aspirin treatment in patients with AMI after PCI was more conducive to myocardial blood flow reperfusion. Studies have pointed out that the combination of ticagrelor and tirofiban had good synergy, which inhibited platelet aggregation from different sites, shortened the effective inhibition of platelet aggregation time, and at the same time, inhibited vascular endothelial damage and cardiomyocyte damage caused by platelet aggregation, reduced slow blood flow, and increased reperfusion levels [22]. Studies have also shown that the combination of the two groups could ameliorate the prognosis of patients after PCI without increasing the incidence of bleeding. It has good clinical effects and safety, which is consistent with our observations [23].

The article "The Clinical Efficacy of Tirofiban Combined with Ticagrelor and Aspirin in Treating Acute Myocardial Infarction by Percutaneous Coronary Intervention and Its Effect on Patients' Cardiac Function" was published in 2022. Journal: J Healthc Eng.

Subsequently, we compared the cardiac function of the two groups of patients before and after treatment as well. The results showed that compared with the control group, LVEF of the joint group was higher, and LVESD and LVEDD were lower, indicating that tirofiban combined with ticagrelor and aspirin treatment could effectively facilitate the AMI patients' cardiac function after PCI compared with ticagrelor and aspirin treatment. Besides, except for a higher platelet count, the joint group had much lower platelet-related parameters, average platelet volume, platelet packing, and platelet volume distribution width than those in the control group. MPV stands for the level of neonatal platelets, which reflects the proliferation of megakaryocytes and platelet production in the bone marrow and is an effective indicator of platelet production speed and platelet activation. An increase in which indicates that the patient is in a thrombotic or prethrombotic state [24]. PDW refers to the dispersion of platelet volume, and its increase indicates that the patient has abnormal platelet aggregation, which can reflect platelet activation more specifically than MPV [25]. Platelet count is an indicator that reflects platelet production and decay, and the change of PCT is generally consistent with the change of platelet count [26]. Studies have shown that tirofiban could reduce the destruction of platelets and the production of larger platelets in patients with AMI, which is conducive to maintaining the stability of platelet count and PCT, thereby preventing thrombosis [27]. At the same time, the combined use of tirofiban with ticagrelor and aspirin could exert a better synergistic effect, improve the clinical thrombolytic effect, and obtain the greatest clinical efficacy through different treatment mechanisms [28].

Studies have shown that inflammatory factors such as TNF-*α* and hs-CRP were involved in the process of atherosclerosis and interact with this process [29]. Our research results show that the treatment of tirofiban combined with ticagrelor and aspirin could effectively and quickly improve the inflammatory response of patients, thereby promoting the recovery of heart function. Finally, to observe the safety of the two medication regimens, we compared the incidence of MACE events and adverse reactions in two groups of patients within three months of treatment. Results showed that the incidence of MACE events in the joint group was notably lower, while there was no obvious difference in terms of adverse reaction incidence between the two groups. Bleeding is normally a problem that needs attention in the treatment of AMI. After PCI, however, tirofiban combined with ticagrelor and aspirin antiplatelet therapy could effectively inhibit platelet aggregation with no fatal or organ dysfunction bleeding occurred. Its incidence of bleeding was of no notable difference with double-antibody treatment, which illustrated that tirofiban combined with ticagrelor and aspirin antiplatelet therapy is of good safety.

The article "The Clinical Efficacy of Tirofiban Combined with Ticagrelor and Aspirin in Treating Acute Myocardial Infarction by Percutaneous Coronary Intervention and Its Effect on Patients' Cardiac Function" was published in 2022. Journal: J Healthc Eng.

## 5. Conclusion

In summary, for patients with AMI undergoing PCI, the application of tirofiban combined with ticagrelor and aspirin could effectively reduce the incidence of no reflow or slow blood flow, improve myocardial perfusion function, and have a significant curative effect. In addition, there is no marked difference in the incidence of adverse reactions between the two regimens, indicating that the triple combination is safer. We will further increase the number of research samples and extend the follow-up time for better clinical results.

## Figures and Tables

**Figure 1:** Comparison of left ventricular function between two groups of patients before and after treatment for 3 months; (a) comparison of LVEF of two groups before and after treatment; (b) comparison of LVEDD of two groups before and after treatment; (c) comparison of LVESD of two groups before and after treatment. ^*∗*^indicates *P* < 0.05.

**Figure 2:** Comparison of serum inflammatory factors before and after treatment between two groups; (a) comparison of hs-CRP before and after treatment between two groups; (b) comparison of TNF-*α* before and after treatment between two groups; (c) comparison of IL-6 before and after treatment between two groups. ^*∗*^indicates *P* < 0.05.

**Table 1:** General information table.

Factors	Joint group *n* = 55	Control group *n* = 47	*t*/*X*^2^	*P*
*Gender*				
Male	31 (56.36)	28 (59.57)	0.107	0.743
Female	24 (43.64)	19 (40.43)		

*Age (years)*				
≥53	27 (49.09)	23 (48.94)	0.001	0.987
<53	28 (50.91)	24 (51.06)		

BMI (kg/m^2^)	22.23 ± 1.22	22.49 ± 1.14	1.106	0.272
*Smoking history*				
Yes	24（43.64）	20 (42.55)	0.012	0.912
No	31（56.36）	27 (57.45)		

*Underlying diseases*				
Hypertension	25 (45.45)	21 (44.68)	0.006	0.938
Hyperlipidemia	22 (40.00)	19 (40.43)	0.002	0.965
Diabetes	32 (58.18)	26 (55.32)	0.085	0.771

*Areas of infarction*				
Anterior wall	25 (45.45)	21 (44.68)	0.102	0.950
Extensive anterior wall	22 (40.00)	20 (42.55）		
Others	8 (14.55)	6 (12.77)		

**Table 2:** Comparison of blood flow grade of TIMI.

Grade	Joint group, n = 55	Control group, n = 47	*X* ^2^	*P*
0 grade	0	3(6.38)	3.617	0.057
1 grade	3(5.45)	14(29.79)	10.80	0.001
2 grade	10(18.18)	10(21.28)	0.154	0.695
3 grade	42(76.36)	20(42.55)	12.15	<0.001

The article "The Clinical Efficacy of Tirofiban Combined with Ticagrelor and Aspirin in Treating Acute Myocardial Infarction by Percutaneous Coronary Intervention and Its Effect on Patients' Cardiac Function" was published in 2022. Journal: J Healthc Eng.

**Table 3:** Comparison of adverse reaction rates between two groups of patients (*n*, (%)).

MACE	Joint group, *n* = 55	Control group, *n* = 47	*X* ^2^	*P*
Cardiac death	0	4(8.51)	—	—
Severe heart failure	1(1.82)	3(6.38)	—	—
Recurrent myocardial infarction	1(1.82)	1(2.13)	—	—
Stent thrombosis	1(1.82)	4(8.51)	—	—
Incidence of MACE	3(5.45)	12(25.53)	8.144	0.004

**Table 4:** Comparison of adverse reaction rates between the two groups of patients (*n*, (%)).

Adverse reactions	Joint group *n* = 55	Control group *n* = 47	*X* ^2^	*P*
General bleeding	3 (5.45)	2 (4.26)	—	—
Heavy bleeding	0	0	—	—
Noncardiogenic dyspnea	2 (3.64)	1 (2.13)	—	—
Gastrointestinal reaction	1 (1.82)	1 (2.13)	—	—
Adverse reaction rate	6 (10.91)	4 (8.51)	0.165	0.685

**Table 5:** Comparison of platelet-related parameters between two groups of patients.

Index	Joint group, *n* = 55	Control group, *n* = 47	*t*	*P*
PLT	202.95 ± 3.52	228.9 ± 5.76	27.88	<0.001
PCT (%)	0.32 ± 0.06	0.22 ± 0.04	9.724	<0.001
PDW (%)	13.68 ± 1.04	10.04 ± 1.09	17.23	<0.001
MPV (fl)	11.66 ± 0.88	8.41 ± 1.13	16.32	<0.001

**Table 6:** Comparison of blood cell-related parameters.

Index	Joint group, *n* = 55	Control group, *n* = 47	*t*	*P*
*RDW*				
Before therapy	11.51 ± 0.94	11.8 ± 0.94	1.553	0.124
After treatment	14.84 ± 1.13	12.94 ± 0.94	9.137	<0.001

*NLR*				
Before therapy	3.55 ± 0.44	3.39 ± 0.45	1.812	0.073
After treatment	2.97 ± 0.53	2.05 ± 0.23	11.04	<0.001

*PLR*				
Before therapy	134.32 ± 7.03	133.73 ± 7.16	0.419	0.676
After treatment	120.67 ± 3.2	128.47 ± 4.87	9.685	<0.001

## Data Availability

The labeled dataset used to support the findings of this study is available from the corresponding author upon request.
